RETRACTED

# The Parenteral Vitamin C Improves Sepsis and Sepsis-Induced Multiple Organ Dysfunction Syndrome via Preventing Cellular Immunosuppression

**DOI:** 10.1155/2017/4024672

**Published:** 2017-01-22

**Authors:** Yu-Lei Gao, Bin Lu, Jian-Hua Zhai, Yan-Cun Liu, Hai-Xia Qi, Ying Yao, Yan-Fen Chai, Song-Tao Shou

**Affiliations:** Department of Emergency Medicine, Tianjin Medical University General Hospital, Tianjin 300052, China

## Abstract

Cellular immunosuppression appears to be involved in sepsis and sepsis-induced multiple organ dysfunction syndrome (MODS). Recent evidence showed that parenteral vitamin C (Vit C) had the ability to attenuate sepsis and sepsis-induced MODS. Herein, we investigated the impact of parenteral Vit C on cellular immunosuppression and the therapeutic value in sepsis. Using cecal ligation and puncture (CLP), sepsis was induced in WT and Gulo^−/−^ mice followed with 200 mg/Kg parenteral Vit C administration. The immunologic functions of CD4^+^CD25^+^ regulatory T cells (Tregs) and CD4^+^CD25^−^ T cells, as well as the organ functions, were determined. Administration of parenteral Vit C per se markedly improved the outcome of sepsis and sepsis-induced MODS of WT and Gulo^−/−^ mice. The negative immunoregulation of Tregs was inhibited, mainly including inhibiting the expression of forkhead helix transcription factor- (Foxp-) 3, cytotoxic T lymphocyte associated antigen- (CTLA-) 4, membrane associated transforming growth factor-*β* (TGF-β^m+^), and the secretion of inhibitory cytokines [including TGF-*β* and interleukin- (IL-) 10], as well as CD4^+^ T cells-mediated cellular immunosuppression which was improved by parenteral Vit C in WT and Gulo^−/−^ septic mice. These results suggested that parenteral Vit C has the ability to improve the outcome of sepsis and sepsis-induced MODS and is associated with improvement in cellular immunosuppression.

## 1. Introduction

Sepsis, which is defined as the life-threatening organ dysfunction caused by the dysregulated host response to infection, is the leading cause of MODS and death among critically ill patients [1–4]. There was a significant loss of immunocytes, mainly including B/T-lymphocytes and gastrointestinal epithelial cells, even at the beginning of sepsis [5–8]. It has been noted that patients gradually enter into a state of immunosuppression after primary hyperinflammatory response, especially cellular immunosuppression, defined as immunoparalysis, which could be a significant cause of the exacerbation of MODS or even death out of sepsis [2, 4]. More and more researches showed that modulating the immunosuppressive stage might be a promising interventional strategy to improve the outcome of sepsis [9]. With sepsis, Tregs subdued the process of inflammation and tissue damage while also causing immune dysfunction, including induction of T-lymphocytic apoptosis, inhibition of CD4^+^/CD8^+^ T-lymphocytic function, and mediation of shifting from the helper T cell (Th) 1 to Th 2 response via the expression of CTLA-4 and TGF-*β*^m+^, as well as anti-inflammatory cytokines (IL-10 and TGF-*β*) [10–15].

RETRACTED

Vit C, characterized as essential endogenous trace element and important physiological antioxidant, is involved in the incidence of sepsis and sepsis-induced MODS, even directly with the survival of septic patients [16, 17]. Vit C is identified as an essential component of the immunological response in humanity and experimental animals which augmented a variety of immune reaction, such as the development of mouse bone marrow derived progenitor cells to functional B/T-lymphocytes, the balance of Th1/Th2 response, and the increased serum levels of IgA and IgM, as well as regulating the balance of proliferation and apoptosis of T cells [18–21]. In addition, treatment with Vit C was correlated with the expression of Foxp-3, the demethylation of Foxp3-TSDR (Treg-specific demethylated region), and the suppressive capacity of Tregs in vitro [22]. Yet, direct effects of Vit C on sepsis-induced cellular immunosuppression are not known. Thus, further investigating the impact of Vit C on sepsis-induced cellular immunosuppression will provide a new evidence for understanding the mechanisms of Vit C in the treatment of sepsis. Humanity completely powerlessly synthesizes Vit C on account of the deficiency of L-gulono-*γ*-lactone oxidase (Gulo), which is the pivotal enzyme in the biosynthesis of Vit C; therefore we conducted studies in transgenic mice lacking Gulo 4 (Gulo^−/−^), to investigate the impact of parenteral Vit C on cellular immunosuppression in sepsis and sepsis-induced MODS.

In the present study, using the classical septic model, that is, CLP, we demonstrated that administration of parenteral Vit C per se markedly improved the outcome of sepsis and sepsis-induced MODS of WT and Gulo^−/−^ mice. The negative immunoregulation of Tregs was inhibited, mainly including decreasing the expression of Foxp-3, CTLA-4, and TGF-*β*^m+^ and the secretion of inhibitory cytokines (TGF-*β* and IL-10), as well as improving CD4^+^ T cells-mediated cellular immunosuppression by parenteral Vit C in WT and Gulo^−/−^ septic mice. These results suggested that parenteral Vit C has the ability to improve the outcome of sepsis and sepsis-induced MODS and associate with improvement in cellular immunosuppression.

## 2. Materials and Methods

### 2.1. Animals

The Gulo^−/−^ C57BL/6J mice were propagated from heterozygous Gulo^+/−^ C57BL/6J mice which were picked up from The Mutant Mouse Regional Resource Center (https://www.mmrrc.org/, No. 000015-UCD) and were maintained on a C57BL/6J background (The Laboratory Animal Center of Chinese Academy of Medical Sciences, number SCXK-Jing-2009-0007, Beijing, China). The WT and Gulo^−/−^ C57BL/6J mice, 6–8 weeks old, 20 ± 2 g, were maintained in a specific pathogen-free condition. They were maintained for about 1 week with Vit C supplementation (3.3 g/L, picked up from Luwei Pharmacy, Jinan, Shan Dong, China) in their drinking water. All procedures were undertaken in accordance with the National Institute of Health Guide for the Care and Use of Laboratory Animal and approved by the Scientific Investigation Board and Tianjin Medical University General Hospital, Tianjin, China.

RETRACTED

### 2.2. Medium and Reagents

The medium was RPMI1640 (Nanjing Keygen Biotech, Nanjing, China) with 10% fetal bovine serum (FBS, Sigma, St. Louis, MO). CD4^+^CD25^+^ Tregs isolation kits were from Miltenyi Biotec GmbH, Bergisch Gladbach, Germany. Cell counting kit-8 (CCK-8) was from Dojindo, Kumamoto, Japan. Fluorescein isothiocyanate- (FITC-) conjugated Annexin-V apoptotic kit, purified hamster anti-mouse CD3/CD28, FITC-conjugated anti-mouse CTLA-4, FITC-conjugated anti-mouse/rat-Foxp-3, and allophycocyanin- (APC-) conjugated anti-mouse/rat-  TGF-*β*^m+^ were from eBioscience, San Diego, CA. ELISA kits for interferon- (IFN-) *γ*, IL-4, IL-10, and TGF-*β* were from Excell Biol, Shanghai, China. Alanine transaminase (ALT), aspartate transaminase (AST), creatinine (Cr), and arterial blood gas (ABG) kits were from Instrumentation Laboratory Company, MA, USA. All primers and SYBR Green Real-Time Polymerase Chain Reaction (RT-PCR) Master Mix were from Applied Biosystems, Carlsbad, CA.

### 2.3. Isolation of Splenic CD4^+^CD25^+^ Tregs and CD4^+^CD25^−^ T Cells

CD4^+^CD25^+^ Tregs and CD4^+^CD25^−^ T cells were isolated using mouse CD4^+^CD25^+^ Tregs isolation kits, which we have recounted [23, 24].

### 2.4. Sepsis Model

 The classical septic model, that is, CLP, is used which we have recounted in our previous studies to induce sepsis [23, 24].

### 2.5. Experimental Design

180 mice were divided into control group (30 mice), WT mice with CLP group [WT (CLP), 50 mice], WT mice with CLP and subcutaneous injection of 200 mg/Kg parenteral Vit C group [WT (CLP + Vit C), 50 mice], Gulo^−/−^ mice with CLP group [Gulo^−/−^ (CLP), 50 mice], and Gulo^−/−^ mice with CLP and subcutaneous injection of 200 mg/Kg parenteral Vit C group [Gulo^−/−^ (CLP + Vit C), 50 mice]. The first administration time of parenteral Vit C was immediately after CLP, and parenteral Vit C was given again after 12 hours. The survival time and rate were recorded for 72 hours in various groups. CD4^+^CD25^+^ Tregs and CD4^+^CD25^−^ T cells were isolated from every group at the point of 24 hours after CLP. The proliferative activity, apoptotic rate, and secretion ability (including IFN-*γ* and IL-4) of CD4^+^CD25^−^ T cells, as well as the expression of Foxp-3, Foxp3-TSDR, Helios, CTLA-4, TGF-*β*^m+^, apoptotic rate, and secretion ability (including IL-10 and TGF-*β*) of CD4^+^CD25^+^ Tregs, were determined. The serum levels of AST, ALT, and Cr, as well as ABG, were determined by The Central Laboratory of Tianjin Medical University General Hospital.

RETRACTED

### 2.6. Flow Cytometric Analysis

The expression levels of Foxp-3, CTLA-4, and TGF-*β*^m+^ of CD4^+^CD25^+^ Tregs, as well as the apoptotic rates of CD4^+^CD25^+^ Tregs and CD4^+^CD25^−^ T cells, were determined by flow cytometer (Becton-Dickinson), which we have recounted [23, 24].

### 2.7. CCK-8 Measurement

The proliferative ability of CD4^+^CD25^−^ T cells was determined by CCK-8, which we have recounted [23, 24].

### 2.8. SYBR Green and Methylation-Sensitive RT-PCR

1 × 10^6^ cells/group were used for distilling the total RNA via the single technique of acid guanidinium thiocyanate-chloroform extraction according to the manufacturer's instruction. The mRNA expressions of Foxp-3, Helios, CTLA-4, TGF-*β*, and IL-10 were tested by SYBR Green RT-PCR. The primer sequences were listed in Table 1. The amplification of PCR consisted of 1 min denaturation step at 95°C followed by 40 cycles of 15 s at 95°C and 40 s at 60°C using the Sequence Detection System (Applied Biosystems). The methylation level of Foxp3-TSDR was determined by Methylation-Sensitive RT-PCR, which has been recounted by Tatura et al. [11]. The primers for Foxp3-TSDR were listed in Table 1.

### 2.9. ELISA Measurement

The levels of IFN-*γ*, IL-4, IL-10, and TGF-*β* were determined by ELISA kits, strictly according to the protocols provided by manufacturer, using microplate reader at OD 450.

### 2.10. Statistical Analysis

Data were represented as mean ± standard deviation (SD) and analyzed by software SPSS 17.0 with one-way ANOVA. Unpaired Student's *t*-test was used to evaluate significant differences between groups. A *p* value of 0.05 or 0.01 was considered statistically significant. Survival rate in septic mice was evaluated by Kaplan-Meier via the log-rank test.

## 3. Results

### 3.1. Parenteral Vit C Improved the Outcome of Sepsis and Sepsis-Induced MODS

As shown in Figure 1(a), compared with WT (CLP) group, the deficiency of Vit C reduced the 72-hour survival rate of Gulo^−/−^ mice (*p* < 0.05); administration of parenteral Vit C significantly increased the survival rate of WT and Gulo^−/−^ mice (*p* < 0.01) in sepsis. Compared with WT (CLP) group at 24 hours after CLP, the deficiency of Vit C worsened the organs function of Gulo^−/−^ (CLP) mice with sepsis, acting as the serum levels of AST (Figure 1(b)), ALT (Figure 1(c)), Cr (Figure 1(d)), and Lac (Figure 1(g)) were elevated, but the levels of PCO_2_ (Figure 1(e)) and PO_2_ (Figure 1(f)) were decreased (*p* < 0.05 or 0.01); administration of parenteral Vit C after CLP significantly improved the appellate quotas of organ function of WT mice and Gulo^−/−^ mice (*p* < 0.05 or 0.01).

RETRACTED

### 3.2. Parenteral Vit C Weakened the Stability of CD4^+^CD25^+^ Tregs with Sepsis

CD4^+^CD25^+^ Tregs were isolated from every group; the deficiency of Vit C inhibited the expression of Foxp-3 (Figure 2(a)), CTLA-4 (Figure 2(b)), and TGF-*β*^m+^ (Figure 2(c)) on splenic CD4^+^CD25^+^ Tregs of Gulo^−/−^ mice (*p* < 0.05 or 0.01), but the expressions of Foxp-3, CTLA-4, and TGF-*β*^m+^ were significantly weakened when parenteral Vit C was administered after CLP to WT mice and Gulo^−/−^ mice (*p* < 0.05 or 0.01).  Figure 2(d) showed that there were no differences between WT and Gulo^−/−^ mice on the apoptotic level of CD4^+^CD25^+^ Tregs, with or without administered parenteral Vit C with sepsis (*p* > 0.05). The supernatant levels of TGF-*β* (Figure 2(e)) and IL-10 (Figure 2(f)) were significantly increased from CD4^+^CD25^+^ Tregs which were isolated from Gulo^−/−^ (CLP) groups after being cultured for 24 hours (*p* < 0.01) but significantly decreased from CD4^+^CD25^+^ Tregs which were isolated from WT and Gulo^−/−^ mice with administration of parenteral Vit C (*p* < 0.05 or 0.01).

### 3.3. Parenteral Vit C Inhibited the Immunosuppressive Function of CD4^+^CD25^+^ Tregs

CD4^+^CD25^+^ Tregs were cocultured with conventional CD4^+^CD25^−^ T cells for another 24 hours in a ratio of 1 : 1 with anti-CD3 (5 *μ*g/mL) and anti-CD28 (2 *μ*g/mL) for polyclonal activation of T cells, respectively. CD4^+^CD25^+^ Tregs which were isolated from Gulo^−/−^ (CLP) group significantly inhibited the proliferative activity (Figure 3(a)) and release of IFN-*γ* (Figure 3(c)) but enhanced the apoptotic rate (Figure 3(b)) and release of IL-4 (Figure 3(d)) of CD4^+^CD25^−^ T cells (*p* < 0.05 or 0.01); however, treatment with parenteral Vit C of WT and Gulo^-/−^ mice significantly inhibited the immunosuppressive function of CD4^+^CD25^+^ Tregs to CD4^+^CD25^−^ T cells which increased the proliferative response and release of IFN-*γ* but decreased the apoptotic rate and release of IL-4 of conventional CD4^+^CD25^−^ T cells (*p* < 0.05 or 0.01).

RETRACTED

### 3.4. The Impact of Parenteral Vit C on the mRNA Expression of Foxp-3, Helios, CTLA-4, TGF-*β*, IL-10, and the Methylation Level of Foxp3-TSDR

The deficiency of Vit C significantly promoted the mRNA expression of* Foxp-3 *(Figure 4(a)),* Helios *(Figure 4(c)),* CTLA-4 *(Figure 4(d)),* TGF-β*  (Figure 4(e)), and* IL-10 *(Figure 4(f)) but decreased the methylation level of* Foxp3-TSDR* (Figure 4(b)) in CD4^+^CD25^+^ Tregs of Gulo^−/−^ (CLP) group in comparison to WT (CLP) group (*p* < 0.01). Treatment with parenteral Vit C after CLP of WT and Gulo^−/−^ mice inhibited the expression of* Foxp-3*,* Helios*,* CTLA-4*,* TGF-β*, and* IL-10* but enhanced the methylation level of* Foxp3-TSDR* in CD4^+^CD25^+^ Tregs (*p* < 0.05 or 0.01).

### 3.5. Parenteral Vit C Improved CD4^+^ T Cells-Mediated Cellular Immunosuppression

CD4^+^CD25^−^ T cells were isolated from every group and cultured for another 24 hours. The deficiency of Vit C significantly worsened the proliferative ability (Figure 5(a)) and IFN-*γ* level (Figure 5(c)) but increased the release of IL-4 (Figure 5(d)) of splenic CD4^+^CD25^−^ T cells of Gulo^−/−^ mice (*p* < 0.01); however, treatment with parenteral Vit C after CLP significantly enhanced the proliferative response and IFN-*γ* level but inhibited the release of IL-4 of CD4^+^CD25^−^ T cells of WT and Gulo^−/−^ mice (*p* < 0.01). As shown in Figure 5(b), the deficiency of Vit C significantly increased the apoptotic rate of splenic CD4^+^CD25^−^ T cells of Gulo^−/−^ mice (*p* < 0.01); however, treatment with parenteral Vit C after CLP decreased the apoptotic rate of CD4^+^CD25^−^ T cells of WT mice and Gulo^−/−^ mice with sepsis (*p* < 0.05 or 0.01).

## 4. Discussion

MODS is the principal cause of death in critically ill patients with sepsis [3]. Fisher BJ and his colleagues showed that low circulatory level of Vit C was significantly susceptible to sepsis-induced MODS [16]. In the current study, we reported that administration of parenteral Vit C per se markedly improved sepsis and sepsis-induced MODS in WT and Gulo^−/−^ mice, which was in accordance with the findings of Fisher BJ. Meanwhile, we first reported the mechanisms of parenteral Vit C in improving the outcome of sepsis and sepsis-induced MODS via regulating cellular immunosuppression.

The immune dysfunction of CD4^+^ T cells is the primary cellular mechanisms with sepsis and sepsis-induced MODS. Immediate specimens from liver, kidney, and lung, even the cellular number of circulatory system in septic patients who died in intensive care units, showed a progressive, profound, apoptosis-induced loss of adaptive immunocytes, especially the early decrease of T-lymphocytes, thereby resulting in an attenuated ability of clearing life-threatening pathogens [2, 5, 7, 8]. The activated CD4^+^ T cells can mainly differentiate into Th1 and Th2 which mainly produced IFN-*γ* and IL-4, respectively. A shift to Th2 response was noted to be corroborated with sepsis-induced MODS and the outcome of sepsis [8, 20, 25, 26]. We showed that administration of parenteral Vit C had the ability to improve the immune dysfunction of CD4^+^ T cells. Sepsis significantly weakened the proliferation and IFN-*γ* secretion but enhanced the apoptotic level and IL-4 secretion of CD4^+^CD25^−^ T cells of WT mice and Gulo^−/−^ mice; however, treatment with 200 mg/Kg parenteral Vit C for two times after CLP significantly took a turn for the better and acted on upregulating the proliferative response and IFN-*γ* secretion as well as downregulating the apoptotic rate and IL-4 secretion. The immunological mechanisms of Vit C on CD4^+^ T cells have not been elucidated; reactive oxygen species (ROS) was formed during CD4^+^ T cells activation which acted as the second messenger [19–21, 27]. We conjectured that parenteral Vit C affects T cell behaviors during sepsis via ROS.

RETRACTED

We have reported that the percentage and stability of Tregs were higher in septic patients than those without sepsis; a reduction in the stability of Tregs was accompanied by an improvement in survival rate and immune dysfunction of T-lymphocytes with sepsis [12–15, 23, 24]. Foxp- 3, which is still the mainly intracellular marker for identification of Tregs, was also critical for their function, differentiation, and maintenance [10, 11]. Our previous study demonstrated that an increased expression of Foxp-3 in Tregs was positively correlated to the mortality of septic mice [12]. Parenteral Vit C weakened the expression of Foxp-3 at protein and gene levels, but the deficiency of Vit C promoted the expression of Foxp-3 in Gulo^−/−^ mice septic model. The recent researches showed that the expression of transcription factor Helios controlled a great deal of pivotal aspects of Tregs' suppressive function, differentiation, and survival [28]. We first reported that sepsis per se promoted the mRNA expression of Helios, especially in the absence of Vit C, but treatment with parenteral Vit C after CLP of WT and Gulo^−/−^ mice inhibited the mRNA expression of Helios. These suggested that parenteral Vit C had significant ability to decrease the stability of Tregs with sepsis.

During the development of sepsis, Tregs can mainly inhibit the activation of CD4^+^ T cells through various mechanisms, mainly including the pathway of cellular contact (e.g., CTLA-4 and TGF-*β*^m+^) and inhibitory cytokines (e.g., IL-10 and TGF-*β*), as well as upregulating the antiapoptotic ability of Tregs [11–15, 23, 24]. Accumulated evidence has shown that a combination of Foxp-3, CTLA-4, TGF-*β*^m+^, and inhibitory cytokines (IL-10 and TGF-*β*) might serve as active markers for Tregs with sepsis. Our previous study demonstrated that sepsis obviously enhanced the negative immunoregulation of Nrp-1^high^CD4^+^CD25^+^ Tregs which correlated to the expression of Foxp-3 and CTLA-4, as well as the secretion of IL-10 and TGF-*β* [23]. We showed that parenteral Vit C could inhibit the expression of exterior CTLA-4 and TGF-*β*^m+^ and the secretion of TGF-*β* and IL-10 at protein and gene levels but did not alter the apoptotic level of CD4^+^CD25^+^ Tregs. These findings were in accordance with the results of our previous studies [12, 13]. The stability of Tregs includes the expression of Foxp-3 and negative immunoregulation with sepsis, which is crucially dependent on the demethylation status of the Foxp3-TSDR [11]. Our previous study suggested that recombinant Nrp-1 polyclonal antibody could decrease the demethylation of Foxp3-TSDR in the presence of LPS, which is associated with inhibition of the negative immunoregulation of Tregs [23]. In the current study, parenteral Vit C had the ability to decrease the demethylation level of Foxp3-TSDR, but the deficiency of Vit C increased the demethylation level of Foxp3-TSDR in Gulo^−/−^ mice septic model, which was in accordance with our previous findings.

RETRACTED

## 5. Conclusion

In conclusion, administration of parenteral Vit C improved the outcome of sepsis and sepsis-induced MODS of WT and Gulo^−/−^ mice. The negative immunoregulation of Tregs was inhibited, mainly including inhibiting the expression of Foxp-3, CTLA-4, and TGF-*β*^m+^ and the secretion of inhibitory cytokines (TGF-*β* and IL-10); CD4^+^ T cells-mediated cellular immunosuppression was improved by parenteral Vit C in WT and Gulo^−/−^ septic mice. These results suggested that parenteral Vit C has the ability to improve the outcome of sepsis and sepsis-induced MODS and is associated with improvement in cellular immunosuppression.

## Figures and Tables

**Figure 1:** The impact of parenteral Vit C treatment on the 72-hour survival rate of septic mice and sepsis-induced MODS. The 72-hour survival rate of WT mice and Gulo^−/−^ mice was improved on administration of 200 mg/Kg parenteral Vit C twice after CLP (a). Parenteral Vit C improved the biomarkers of liver (b and c), renal (d), respiratory (e and f), and circulatory (g) function in CLP-exposed WT mice and Vit C deficient Gulo^−/−^ mice. The survival rate was analyzed by Kaplan-Meier via the log-rank test, *n* = 50 per group. WT (CLP) versus WT (CLP + Vit C), *p* < 0.01. Gulo^−/−^ (CLP) versus Gulo^−/−^ (CLP + Vit C), *p* < 0.01. WT (CLP) versus Gulo^−/−^ (CLP), *p* < 0.05. Data were represented as mean ± standard deviation (SD) and analyzed by software SPSS 17.0 with one-way ANOVA, *n* = 4 per group, ^*∗*^*p* < 0.05 or ^*∗∗*^*p* < 0.01.

RETRACTED

**Figure 2:** Parenteral Vit C markedly weakened the stability of CD4^+^CD25^+^ Tregs in sepsis. The expressions of Foxp-3, CTLA-4, and TGF-*β*^m+^, as well as the apoptotic ability of splenic CD4^+^CD25^+^ Tregs, were subjected to flow cytometric analysis by flow cytometer (g). Parenteral Vit C downregulated the expression of Foxp-3 (a), CTLA-4 (b), and TGF-*β*^m+^ (c) of CD4^+^CD25^+^ Tregs in sepsis. Parenteral Vit C did not alter the apoptotic ability of splenic CD4^+^CD25^+^ Tregs in sepsis (d). Parenteral Vit C inhibited the secretion of TGF-*β* (e) and IL-10 (f) from CD4^+^CD25^+^ Tregs in sepsis. Data were represented as mean ± standard deviation (SD) and analyzed by software SPSS 17.0 with one-way ANOVA, *n* = 4 per group, ^*∗*^*p* < 0.05 or ^*∗∗*^*p* < 0.01.

**Figure 3:** The impact of parenteral Vit C on the immunosuppressive function of CD4^+^CD25^+^ Tregs. The parenteral Vit C inhibited the immunosuppressive function of CD4^+^CD25^+^ Tregs which upregulated the proliferative response (a) and release of IFN-*γ* (c) but significantly downregulated the apoptotic rate (b) and release of IL-4 (d) of splenic conventional CD4^+^CD25^−^ T cells. Data were represented as mean ± standard deviation (SD) and analyzed by software SPSS 17.0 with one-way ANOVA, *n* = 4 per group, ^*∗*^*p* < 0.05 or ^*∗∗*^*p* < 0.01.

**Figure 4:** The impact of parenteral Vit C on the mRNA expression of* Foxp-3*,* Helios*,* CTLA-4*,* TGF-β*,* IL-10*, and the methylation level of* Foxp3-TSDR* mRNA in CD4^+^CD25^+^ Tregs; CD4^+^CD25^+^ Tregs were harvested for SYBR Green and Methylation-Sensitive RT-PCRT from every group after CLP. The parenteral Vit C inhibited the expression of* Foxp-3 *(a),* Helios *(c),* CTLA-4 *(d),* TGF-β*  (e), and* IL-10 *(f) but increased the methylation level of* Foxp3-TSDR* (b) in CD4^+^CD25^+^ Tregs. Data were represented as mean ± standard deviation (SD) and analyzed by software SPSS 17.0 with one-way ANOVA, *n* = 4 per group, ^*∗*^*p* < 0.05 or ^*∗∗*^*p* < 0.01.

**Figure 5:** The impact of parenteral Vit C on CD4^+^ T cells-mediated cellular immunosuppression in sepsis. Treatment with 200 mg/Kg parenteral Vit C upregulated the proliferative response of CD4^+^CD25^−^ T cells of WT mice and Gulo^−/−^ mice in sepsis (a). The apoptotic rate of splenic CD4^+^CD25^−^ T cells was analyzed with Annexin-V-FITC/PI by flow cytometry at 24 hours after CLP-induced midgrade sepsis (e). The apoptotic level of splenic CD4^+^CD25^−^ T cells was decreased when 200 mg/Kg parenteral Vit C was administered after CLP to WT mice and Gulo^−/−^ mice in sepsis (b). Parenteral Vit C increased the serum level of IFN-*γ* (c) as well as decreasing the serum levels of IL-4 (d) of WT mice and Gulo^−/−^ mice in sepsis. Data were represented as mean ± standard deviation (SD) and analyzed by software SPSS 17.0 with one-way ANOVA, *n* = 4 per group, ^*∗*^*p* < 0.05 or ^*∗∗*^*p* < 0.01.

RETRACTED

**Table 1:** Targeted genes and their primer sequences for SYBR Green and Methylation-Sensitive Real-Time Polymerase Chain Reaction.

Gene	Primer sequences
Mouse Foxp-3	Forward: 5′-CAGCTGCCTACAGTGCCCCTAG-3 Reverse: 5′-CATTTGCCAGCAGTGGGTAG-3′
Mouse Helios	Forward: 5′-TAAGCTCAGCTTATTCTCAGGTCTATCA-3′ Reverse: 5′-ATGTTGTTTTCGTGACTATCAGATGTT-3′
Mouse CTLA-4	Forward: 5′-CGCAGATTTATGTCATTGATCC-3′ Reverse: 5′-TTTTCACATAGACCCCTGTTGT-3′
Mouse TGF-*β*	Forward: 5′-AACAATTCCTGGCGTTACCTT-3′ Reverse: 5′-GAATCGAAAGCCCTGTATTCC-3′
Mouse IL-10	Forward: 5′-ACAGCCGGGAAGACAATAAC-3′ Reverse: 5′-CAGCTGGTCCTTTGTTTGAAAG-3′
Mouse Foxp3-TSDR	Forward: 5′-CTTGCTTCCTGGCACGAGATTTGAATTGGATATGGTTTGT-3′ Reverse: 5′-CAGGAAACAGCTATGACAACCTTAAACCCCTCTAACATC-3
